The article "The Impact of 3S2E Nursing Management on the Psychological Status of Respiratory Function and Quality of Life of Patients with Severe Pneumonia in the ICU" was retracted in 2023. Reasons: signs of a paper mill; compromised peer review; unreliable results or conclusions.

# The Impact of 3S2E Nursing Management on the Psychological Status of Respiratory Function and Quality of Life of Patients with Severe Pneumonia in the ICU

**DOI:** 10.1155/2022/4949498

**Published:** 2022-09-23

**Authors:** Yaoyao Xu, Xia Li, Qin Yang, Xiuxian Ma

**Affiliations:** Department of Critical Care Medicine, Traditional Chinese Medicine, Wenzhou Municipal Hospital of Traditional Chinese Medicine, Wenzhou 325000, China

## Abstract

**Objective:**

This study examines the effects of the 3S2E nursing management mode on patients with severe pneumonia in the intensive care unit's respiratory function, psychological status, and quality of life (ICU).

**Methods:**

According to a random number table, 82 ICU patients with severe pneumonia who were admitted between March 2021 and March 2022 were enrolled and assigned to the control and observation class (*n* = 41, respectively) in a 1 : 1 ratio. The observation class added 3S2E manner in addition to ordinary breastfeeding, whereas the control class received treatment in the usual nursing mode. The two groups' preintervention and postintervention times for mechanical ventilation, white blood cell count (WBC) recovery, duration of hospital stay, problems, respiratory function, psychological state, and living quality were compared.

**Results:**

Fever time abatement, mechanical ventilation time, WBC recovery time, and length of hospital stay in the observation category were found to be shorter in comparison with the control class (*P* < 0.05). In contrast to the other group, the observation group had fewer issues (*P* < 0.05). Both teams' oxygenation indices and SaO_2_ were higher after the intervention (*P* < 0.05), with the observation team's index being higher than the control group's index. The total SAS and SDS scores of the two groups were less in the postintervention period than in the preintervention period, with the observational class having lower postintervention SAS and SDS ratings than the comparison group (*P* < 0.05). The postintervention ratings in the observation class were higher than those in the control, and the World Health Organization Quality of Life (WHOQOL) scale scores in the 2 categories were greater after the intervention than they were before (*P* < 0.05).

**Conclusion:**

3S2E nursing management model improves respiratory function, alleviates negative emotions, and improves living quality in ICU patients with severe pneumonia.

## 1. Introduction

Pneumonia is one of the commonest infections in elderly patients. The major cause of mortality in pneumonia is lower respiratory tract infection. Pneumonia in the elderly is mostly correlated with age-dependent and pathologic changes in the immune system and the lungs. 3S2E nursing management is a new nursing management model based on nursing safety systems and clinical practices, which has achieved a good effect on severe diseases in recent years.

A common respiratory condition that requires special treatment is severe pneumonia. The patient's lung tissue develops from acidosis, hypoxia, and viral and bacterial attack, which usually affects multiple organs [1–3]. Severe pneumonia may progress to multiple organ dysfunction syndromes and septic shock, and the disease is life-threatening with high mortality, which requires timely and effective treatment [4, 5]. At present, the treatment plan and nursing intervention for severe pneumonia still need to be improved, and effective nursing intervention is particularly critical for the rehabilitation of patients [2, 6]. The intervention of “3S2E” nursing management model in patients with severe pneumonia can improve the patient's respiratory function and reduce their anxiety and depression [1, 7]. Therefore, this study focused on 3S2E on respiratory function, psychological health, and standard of living of ICU patients with severe pneumonia.

This study aimed to demonstrate the role of 3S2E nursing management model in respiratory function living quality in ICU patients with severe pneumonia.

## 2. Data and Methods

### 2.1. Objects and Groups

According to a random number table, 82 ICU individuals with severe pneumonia who were admitted between June 2021 and June 2022 were enrolled and assigned to the control class and observation class (*n* = 41, respectively) in 1 : 1 ratio. In the control group, there were 25 men and 16 women, respectively, and the weight ranged from 43 to 82 kg, with an average of 62.34 ± 8.85 kg; the average age was 71.64 6.94 years. The observation group consisted of 24 men and 17 women. The average age was 72.02 ± 7.94, with a range of 60 to 86 years. Between 41 and 87 kg, the average weight was 63.42 ± 9.29 kg. The baseline data did not significantly differ between both categories (*P* > 0.05).

### 2.2. Inclusion and Exclusion Criteria

#### 2.2.1. Inclusion Criteria

(1) It was built on 2007 [6] Infectious Diseases Society of America/American Thoracic Society diagnostic criteria for severe pneumonia; (2) the patient has normal cognitive function and communication abilities; (3) the form of informed consent was signed by the patient.

#### 2.2.2. Exclusion Criteria

(1) Those having autoimmune diseases/tumors; (2) pulmonary diseases other than severe pneumonia; (3) the liver and kidney function of the patient was severely impaired; (4) those with cognitive dysfunction or severe mental illness; (5) patients with other severe infections.

### 2.3. Participants

The control group applied routine nursing management, which included the following (1) psychological intervention: medical staff communicate with sufferers to understand their psychological status, carried out individualized psychological intervention according to the psychological characteristics of patients, and told successful cases for fearful and pessimistic patients. Patients with anxiety and depression can be adjusted by listening to music for relief to improve their confidence in treatment. (2) Respiratory care: for patients with mechanical ventilation, the humidification of their airway should be ensured to avoid pipe blockage. For patients who were unable to expectorate, the sputum should be discharged through postural drainage. The patients with thick sputum were treated by atomization inhalation to expel the sputum. (3) Oxygen therapy care: patients with carbon dioxide retention should carry out low-flow uninterrupted oxygen inhalation, and the oxygen concentration needs to be kept at 30%–35%. For patients with hypoxic symptoms, their blood oxygen saturation should be closely monitored, and appropriate oxygen inhalation methods should be used to keep the patient's oxygen flow at 5 L/min. (4) Management of complications: as severe pneumonia is prone to multiple complications, the complications should be reported and handled in time.

Our study was approved by the institutional review board of the hospital and was conducted in accordance with the ethical principles of Helsinki. Written informed consent was obtained from each participant.

Based on the usual nursing care provided to the control group, the observational class was given care using the 3S2E nursing management method. A 3S2E nursing team consisting of a leading physician, a leading nurse, a head nurse, and a nurse was set up, and the detailed management methods were as follows: (1) S1 (improvement of nursing skills): provided standardized training for nurses, including how to dynamically observe the patient's condition, detect abnormalities in time, and maintain effective venous access. All nurses learned the latest disease-related knowledge, nursing progress, and surgical knowledge and carried out nursing skills assessment, and for those who fail the assessment, multiple pieces of training were required to improve their nursing skills. (2) S2 (optimization of nursing services): the basic services should be consolidated, and basic nursing measures should be implemented accordingly. The nursing staff should provide humanistic care to patients and meet their reasonable needs as far as possible in order to provide patients with a good inpatient environment. More communication should be conducted with patients to relieve their negative emotions. The changes of blood oxygen saturation, blood pressure, and inflammatory factors of patients were recorded and evaluated to formulate targeted monitoring and rehabilitation programs. (3) S3 (ensuring safe nursing care): medical staff should prepare risk prevention plans and receive training in advance, especially guidance on key procedures such as catheterization, intubation, and sputum aspiration, so as to ensure the safe transfer and transfer of patients and standardize the rational use of drugs. (4) E1 (evaluation): the medical staff assessed the patient's respiratory function such as oxygenation index and SaO2. (5) E2 (health education): following patient's hospitalization, the responsible nurse introduced the ward and hospital environment to his family members and distributed disease knowledge brochures. Health education was conducted according to patients' different personalities and education levels, including knowledge related to severe pneumonia, treatment methods, family care, and successful case analysis. At least 15 minutes of mental health education should be given to enhance their confidence.

### 2.4. Observation of Indicators

(1) The antipyretic time, mechanical ventilation time, WBC recovery time, and hospital stay of the two groups were observed. (2) The two groups' complications were noticed. (3) Before and following the intervention, alterations in the respiratory function indices, including the oxidation index and SaO_2_, were seen in the two groups. (4) Monitoring the two groups' psychological states before and after the intervention. To assess anxiety and depression, respectively, the Self-Rating Anxiety Scale (SAS) and Self-rating Depression Scale (SDS) were employed. The more severe the patients' anxiety or sadness, the higher the score. (5) Pre- and postintervention observations revealed changes in four different aspects of quality of life, including the environment, social relationships, psychology, and physiology. Each factor was translated to a scale of 100, with higher scores indicating better life quality.

### 2.5. Statistical Treatment

Data processing was conducted by SPSS 26.0. The counting data were expressed as *n* (%) and were subjected to a *t*-test analysis for the measuring data. When *P* < 0.05, the difference was significant.

## 3. Results

### 3.1. Comparison of the Length of Hospital Stay, Mechanical Ventilation, WBC Recovery, and Time for Fever Abatement

In comparison with the control group, the observation group's length of hospital stay, length of mechanical ventilation, recovery of WBC, and time from fever were all shorter (*P* < 0.05) (Table 1).

### 3.2. Comparison of Complications

Fewer complications occurred in the observation group compared to the control group (*P* < 0.05) (Table 2).

### 3.3. Comparison of Respiratory Function

Following the intervention, both groups' oxygenation index and SaO_2_ levels were higher than they had been previously (*P* < 0.05); the monitoring unit had greater indications than the control (*P* < 0.05) (Table 3).

### 3.4. Psychological Status Comparison

The two groups postintervention SAS and SDS scores were lower than their preintervention scores (*P*0.05); the observation group's postintervention SAS and SDS scores were lower than those of the control group's (*P* < 0.05) (Table 4 and Figure 1).

### 3.5. WHOQOL-BREF Comparison

The postintervention World Health Organization Quality of Life (WHOQOL) scores in the observation group were greater than those in the control group (*P* < 0.05), and the scores in the two groups after the intervention were better than those before the intervention (Table 5).

## 4. Discussion

Atypical pneumonia is caused by atypical pathogens that are not detectable with Gram stain and cannot be cultured using standard methods. Severe pneumonia has an acute onset and rapid progress and is often accompanied by varying degrees of respiratory failure, septic shock, and decreased blood pressure. Excitation of the sympathetic adrenal concomitant system results in decreased intestinal perfusion pressure and vasoconstriction of the intestinal mucosa, which then leads to ischemia and hypoxia of intestinal mucosal tissues [7, 8]. In addition, severe pneumonia is in a negative nitrogen balance, which leads to a decline in the patient's immune status. The increased permeability of the intestinal mucosa and the impaired barrier function will aggravate the systemic inflammatory response, thus forming a vicious circle and leading to the occurrence of multiple organ dysfunction syndromes [9–11]. Prompt and effective treatment and nursing are of great significance to severe pneumonia. With the ceaseless changes in medical models and the gradual increase in patients' demand for nursing care, traditional routine care has been unable to meet the needs of patients [12–15]. Therefore, a new nursing model that is promoted for people with severe pneumonia is quite significant.

3S2E nursing management mode is a new nursing mode. It primary enhances nursing service awareness, improves nursing skills, ensures nursing safety, evaluates patients' conditions, and provides health education for them [16–19]. In the 3S2E nursing management mode, nursing staff provide high-quality nursing services for patients, focus on the changes in patient's vital signs, and inform physicians in time when abnormal conditions are found, to facilitate timely treatment by physicians and ameliorate patients' prognosis. This study put forward the fever abatement time and mechanical ventilation. Patients in the observation category had shorter hospital stays and WBC recovery than those in the control category. It considered that the 3S2E nursing management mode can speed up the patient's fever reduction and WBC recovery and can shorten mechanical ventilation time and hospitalization. The nurse management approach was able to lower the occurrence of complications as evidenced by the fact that the complications in the observation group were lower than those in the control group. After the intervention, the patients in the observation group had greater SaO_2_ and oxygenation indices than the patients in the control group, suggesting that the nurse management approach might aid patients with their respiratory function. After the intervention, the SAS and SDS scores of the patients in the observation class were less than those in the control category, suggesting that the psychological status of patients can be improved through the 3S2E nursing management mode. The reason may be that this nursing mode adopted varying forms of intervention, and nursing staff could focus on patients' psychological feelings, which can more effectively improve the psychological state of patients. Following the intervention, the WHOQOL-BREF ratings in the observation category were higher than those in the control group, indicating that the 3S2E nursing management might enhance patients' quality of life. The analysis showed that the physiology and psychology of the human body are integrated and interact with each other, and the living quality can be guaranteed by improving their psychological state.

## 5. Conclusion

In summary, the 3S2E nursing management model improves respiratory function, alleviates negative emotions, and improves living quality in ICU patients with severe pneumonia.

## Figures and Tables

**Figure 1:** Comparison of psychological status (a): SAS scores of the two groups in post-intervention were less than in pre-intervention, the observation group had lower post-intervention SAS than the control group; (b): SDS scores of the two groups in post-intervention were less than in pre-intervention, the observation group had lower post-intervention SDS than the control group. compared with pre-intervention ^*∗*^*P* < 0.05. compared with the control group, ^#^*P* < 0.05.

**Table 1:** Comparison of the two groups' hospital stays, WBC recovery times, mechanical ventilation times, and times for fever abatement ($\bar{x}\pm s$, d).

Group	Number of cases	Time of fever abatement	Mechanical ventilation	WBC recovery	Length of hospital stay
Observation group	41	5.45 ± 1.42	6.23 ± 1.46	6.54 ± 1.38	20.47 ± 5.46
Control group	41	8.37 ± 1.71	9.28 ± 2.35	9.74 ± 1.64	29.38 ± 4.58
*t*		8.412	7.059	9.560	8.006
*P*		<0.05	<0.05	<0.05	<0.05

**Table 2:** Complications comparison.

Group	Number of cases	Bronchiectasis	Pulmonary edema	Septic shock	Incidence (%)
Observation group	41	1	1	1	7.32
Control group	41	5	3	3	26.83
*t*					5.513
*P*					<0.05

**Table 3:** Comparison of respiratory function ($\bar{x}\pm s$).

Group	Number of cases	Oxygenation index (mmHg)		SaO_2_ (%)	
		Pre-intervention	Post-intervention	Pre-intervention	Post-intervention
Observation group	41	217.95 ± 14.32	285.32 ± 22.41^*∗*^	83.24 ± 2.51	96.87 ± 2.18^*∗*^
Control group	41	215.62 ± 18.85	250.87 ± 17.89^*∗*^	83.61 ± 2.37	92.17 ± 2.43^*∗*^
*t*		0.630	7.693	0.686	9.219
*P*		>0.05	<0.05	>0.05	<0.05

*Note.* compared with pre-intervention ^*∗*^*P* < 0.05.

**Table 4:** Psychological status comparison ($\bar{x}\pm s$, points).

Group	Number of cases	SAS		SDS	
		Pre-intervention	Post-intervention	Pre-intervention	Post-intervention
Observation group	41	64.35 ± 4.51	44.52 ± 4.17^*∗*^	61.48 ± 3.47	43.61 ± 3.27^*∗*^
Control group	41	62.79 ± 5.12	49.87 ± 3.68^*∗*^	62.08 ± 3.65	48.42 ± 4.56^*∗*^
*t*		1.464	6.160	0.763	5.489
*P*		>0.05	<0.05	>0.05	<0.05

*Note.* compared with pre-intervention ^*∗*^*P* < 0.05.

**Table 5:** WHOQOL-BREF comparison ($\bar{x}\pm s$, points).

Group	Number of cases	Environment		Social		Psychological field		Physical field	
		Pre-intervention	Post-intervention	Pre-intervention	Post-intervention	Pre-intervention	Post-intervention	Pre-intervention	Post-intervention
Observation group	41	52.35 ± 5.35	73.24 ± 3.56^*∗*^	70.64 ± 4.26	87.87 ± 4.49^*∗*^	44.52 ± 5.41	70.25 ± 5.67^*∗*^	47.42 ± 5.67	76.52 ± 4.58^*∗*^
Control group	41	53.24 ± 4.26	64.51 ± 4.78^*∗*^	72.01 ± 3.89	81.02 ± 5.45^*∗*^	43.78 ± 3.54	61.98 ± 4.72^*∗*^	48.18 ± 5.25	63.37 ± 5.07^*∗*^
*t*		0.833	9.379	1.521	6.212	0.733	7.178	0.630	12.324
*P*		＞0.05	＜0.05	＞0.05	＜0.05	＞0.05	＜0.05	＞0.05	＜0.05

*Note.* compared with pre-intervention ^*∗*^*P* < 0.05.

## Data Availability

The data used to support this study is available from the corresponding author upon request.
